# SKA1 promotes malignant phenotype and progression of glioma via multiple signaling pathways

**DOI:** 10.1186/s12935-019-1047-z

**Published:** 2019-12-03

**Authors:** Xizhao Wang, Yu Zeng, Mingfeng Zhou, Xian Zhang, Anqi Xu, Jie Lin, Zhiyong Wu, Cheng Xie, Jie Luo, Shengfeng Ding, Zhengming Zhan, Hao Long, Ye Song

**Affiliations:** 1 Department of Neurosurgery, Nanfang Hospital, Southern Medical University, Guangzhou, 510515 Guangdong People’s Republic of China; 2 Department of Neurosurgery, The First Hospital of Quanzhou Affiliated to Fujian Medical University, Quanzhou, 362000 Fujian People’s Republic of China; 3 Department of Neurosurgery, Shanghai Tenth People’s Hospital, Tongji University School of Medicine, Shanghai, 200072 People’s Republic of China

**Keywords:** SKA1, Glioma, Malignant phenotype, Cell cycle, EMT, Wnt/β-catenin signaling pathway

## Abstract

**Background:**

Spindle and kinetochore associated protein 1 (SKA1) is a protein involved in chromosome congression and mitosis. It has been found to be upregulated and oncogenic in several human cancers. Herein, we investigated the precise role of SKA1 in the progression and malignant phenotype of human glioma.

**Methods:**

Bioinformatic analysis was carried out based on the RNA-seq data and corresponding clinical data from GEO, TCGA and CGGA databases. Western blot was performed to analyze the expression of SKA1 in clinical samples and signaling pathway proteins in glioma cells, respectively. CCK8 assay, colony forming assay and EdU assay were performed to assess the cell viability. Cell migration and invasion assays were also performed. Moreover, xenograft model was established and the expression of SKA1 was assessed in the xenograft by immunohistochemistry.

**Results:**

SKA1 expression is positively correlated with glioma grade and could be a promising biomarker for GBM. Moreover, overexpression of SKA1 may lead to poor prognosis in glioma. Downregulation of SKA1 attenuated cell viability, migration, and invasion in U251, U87, LN229 and T98 cells. Furthermore, GSEA analysis demonstrated that SKA1 was involved in the cell cycle, EMT pathway as well as Wnt/β-catenin signaling pathway, which were then confirmed with Western blot analysis.

**Conclusion:**

SKA1 promotes malignant phenotype and progression of glioma via multiple pathways, including cell cycle, EMT, Wnt/β-catenin signaling pathway. Therefore, SKA1 could be a promising therapeutic target for the treatment of human gliomas.

## Background

Gliomas are the most common primary tumors in the central nervous system in adults, with an estimated annual incidence of 6.6 per 100,000 individuals in the USA [1]. Glioblastoma is the most malignant type of glioma and leads to poor survival despite of aggressive therapy including surgery, radiotherapy and chemotherapy [2–5]. The 2016 WHO classification of tumors of the central nervous system proposed the priority of integrated histological and molecular classification system in brain tumor diagnosis, which enables more precise patient stratification [1]. It is indicated that glioblastoma patients with different recurrence-free survival (RFS) time exhibited different expression pattern of mRNAs and miRNAs [6]. Considering the heterogeneity within and among glioma patients, more insights into the oncogenes of glioma are still an urgent need.

Spindle and kinetochore associated complex (SKA complex) is required for timely anaphase onset. This family is composed of three proteins: SKA1, SKA2 and SKA3, which facilitates the processive movement of microspheres along with depolymerizing microtubules. Individually, SKA1 complex mostly performed two crucial biochemical functions: direct microtubule binding through its C-terminal domain, and microtubule-stimulated oligomerization [7, 8]. Inhibition of the SKA complex results in a chromosome congression failure followed by cell death [9–12]. The role of SKA1 in the malignant progression of several cancers has already been discussed recently [13–16]. In vitro experiments revealed that SKA1 may be a potential therapeutic target of human glioblastoma [17], but the underlying mechanisms remains to be elucidated.

Here, we confirmed that expressions of SKA1 increased along with advances in glioma grades. Knockdown of SKA1 could potently inhibit proliferation, migration and invasion both in vitro and in vivo. We further clarified that SKA1 was involved in Wnt/β-catenin signaling pathway and could be a potential biomarker of malignant phenotype in glioma.

## Methods

### Bioinformatic analysis

Data used in this study for bioinformatic analysis was obtained from public datasets, including GEO Datasets (https://www.ncbi.nlm.nih.gov/gds/), TCGA (https://cancergenome.nih.gov/) and CGGA (http://www.cgga.org.cn/). Gene set enrichment analysis (GSEA) was further performed to explore the potential roles of SKA1.

### Cell culture

The human glioma cell lines U251, U87, LN229 and T98 were purchased from the Chinese Academy of Sciences (Shanghai, China). In the laboratory, all cell lines were grown in Dulbecco’s modified Eagle’s medium (DMEM) (Hyclone, Logan, UT) supplemented with 10% fetal bovine serum (FBS, Hyclone, Logan, UT) and incubated in a humidified atmosphere of 5% CO_2_ at 37 °C.

### Clinical tissue sample collection

Tumor tissues were collected from patients with pathologically and clinically confirmed glioma. All samples were confirmed by pathological diagnosis and classified according to the World Health Organization (WHO) criteria. Moreover, prior written informed consents were obtained from patients or their guardians, and approval from the Ethics Committees of Nanfang Hospital of Guangdong Province were also obtained.

### Establishment of stably transfected cells

The preparation of lentivirus expressing human SKA short hairpin RNA (sh#1, CCGGTGAAGAACCTGAACCCGTAAACTCGAGTTTACGGGTTCAGGTTCTTCATTTTTTG; sh#2, CCGGATAGAGTATAGAGGCTATTTCCTCGAGGAAATAGCCTCTATACTCTATTTTTTTG; sh#3, CCGGCCTGACACAAAGCTCCTAAATCTCGAGATTTAGGAGCTTTGTGTCAGGTTTTTG) were performed using the pLVTHM-GFP lentiviral RNAi expression system (Genechem, China). U87, U251, LN229 and T98 cells were then transfected with lentiviral particles containing specific or negative-control (shNC) vectors according to the manufacturer’s instructions, respectively.

### Western blot analysis

The cells or tumor tissues were washed three times with PBS and lysed in RIPA Buffer (50 mM Tris–HCl pH 8.0, 1 mM EDTA pH 8.0, 5 mM DTT, 2% SDS) with protease inhibitor and phosphoric-acid protease inhibitor at 4 °C for 30 min. Then they were crushed with ultrasonic machine and centrifuged at 12000 rpm for 15 min at 4 °C. The protein concentration was measured using BCA assay (Beyotime Inc, China). 12.5 μl mixed solution including 30 mg protein and 2.5 μl SDS was resolved using a 10% SDS-PAGE gel and electro-transferred to polyvinylidene fluoride membranes (Invitrogen, Carlsbad, CA). Afterwards, the membranes were blocked with 5% BSA or nonfat milk in pH 7.0 TBST, and then were incubated with primary antibodies overnight at 4 °C. On the next day, membranes were washed three times with TBST and incubated with horseradish peroxidase conjugated secondary antibody for 1 h at room temperature. At last, membranes were washed three times with TBST again. Signals were detected using enhanced chemiluminescence reagents (Pierce, Rockford, IL, USA). All experiments were independently performed in triplicate.

### CCK8 assay

The CCK8 assay was performed to examine cell viability. Glioma cells (1000/well) were seeded in 96-well plates with a volume of 200 μl medium. Subsequently, 10 μl of CCK8 reagent mixed with 100 μl DMEM medium without FBS were added to each well and incubated for 1 h. Then the absorbance value (OD) was measured at 450 nm. The observation duration lasted for one week at the same time every day.

### Colony forming assay

The indicated cells were plated in 12-well plates (200 cells per well) and cultured for 2 weeks. The colonies were then fixed with methanol for 30 min and stained with 1% crystal violet for 1 min. All assays were independently performed in triplicate.

### EdU incorporation assay

The proliferation of U87 and U251 cells were examined using the Cell-Light EdU Apollo488 In Vitro Imaging Kit (RiboBio, China) according to the manufacturer’s protocol. In brief, cells were incubated with 10 μM EdU for 2 h before fixation with 4% paraformaldehyde and permeabilization with 0.5% Triton X-100, and then stained with EdU kit. Cell nucleus were stained with 5 μg/ml DAPI (4′,6-diamidino-2 phenylindole) for 10 min. The number of EdU-positive cells was counted under a microscope in five random fields (200×). All assays were independently performed in triplicate.

### Cell migration and invasion assay

The cell migration assays were carried out with Transwell assays. About 5 × 10^4^ cells in 100 μl DMEM medium without FBS were seeded on a fibronectin-coated polycarbonate membrane inserted in a Transwell apparatus (Costar, MA). In the lower chamber, 500 μl DMEM with 10% FBS was added as a chemoattractant. After the cells were incubated for an appropriate time according to specific cell lines in a 5% CO_2_ atmosphere at 37 °C, the insert was washed with PBS, and cells on the top surface of the insert were removed with a cotton swab. Cells adhering to the lower surface were fixed with methanol for 30 min, stained with 1% crystal violet solution for 1 min and counted under a microscope in three random fields. The cell invasion assays were carried out with Boyden assays, and the procedure was similar to the cell migration assay, except for that polycarbonate membranes were precoated with 24 mg/ml Matrigel (R&D Systems, USA). All assays were independently performed in triplicate.

### Wound healing assay

U87 and U251 cells were stably transfected with shSKA1 or empty vectors respectively, and then cultured in 6-well plates. After the cells grew to 90% confluence, three paralleled scratch wounds across each well were made with a P-10 pipette tip. Fresh medium supplemented with reduced FBS (5%) was added, and the wound-closing procedure was observed for 48 h. Photographs were taken at 0, 12 h, 24 h and 48 h, respectively. All assays were independently performed in triplicate.

### Xenograft tumor model

About 1 × 10^6^ active U87 cells that transfected with shRNA or empty vectors and suspended in 0.1 ml DMEM medium were subcutaneously injected into a group of ten nude mice, respectively. These mice were grown in a barrier facility on HEPA-filtered racks. The animals were fed with an autoclaved laboratory rodent diet and water. All animal studies were conducted in accordance with the principles and procedures outlined in the National Institutes of Health Guide for the Care and Use of Animals under assurance number A3873-1. On day 30, the mice were sacrificed, and tumor tissues were excised and weighed, respectively.

### Immunohistochemistry

Paraffin sections at 4 μm were deparaffinized in 100% xylene and rehydrated in descending ethanol series according to standard protocol. Heat-induced antigen retrieval was performed in citrate buffer for 15 min in microwave oven. Endogenous peroxidase activity and non-specific antigens were blocked with peroxidase blocking reagent containing 3% hydrogen peroxide and serum. The sections were then incubated with primary antibodies, including N-cadherin (1:100; CST, USA), E-cadherin (1:100; Proteintech, USA), MMP9 (1:100; Proteintech, USA), and PCNA (1:100; Abcam, USA), at 4 °C overnight. The next day, the sections were washed three times with PBS. The sections were followed by incubation with biotin-labeled secondary antibody for 1 h at room temperature and washed three times with PBS. Subsequently, Sections were visualized with DAB and counterstained with hematoxylin, mounted in neutral gum, and analyzed with a bright field microscope equipped with a digital camera (Nikon, Japan). The results were scored as previously mentioned: 0, no staining; 1, weak staining in < 50% cells; 2, weak staining in ≥ 50% cells; 3, strong staining in < 50% cells; and 4, strong staining in ≥ 50% cells [18]. All experiments were independently performed in triplicate.

### Statistical analysis

All quantified data is presented as an average of triplicate technical replicates. SPSS 13.0 and Graph Pad Prism 4.0 software were used for statistical analysis. Data are represented as mean ± SD. One-way ANOVA or two-tailed Student’s t-test was used for comparisons between groups. Chi square test or Fischer’s were used to identify differences between categorical variables. Survival analysis was performed using Kaplan–Meier method. Multivariate Cox proportional hazards method was used for analyzing the relationship between the variables and patient’s survival status. Differences were considered statistically significant when P < 0.05.

## Results

### SKA1 expression was positively associated with glioma grade

First, SKA1 expression was determined in public data deposited in TCGA database and GEO dataset (GSE 4290). We found that SKA1 expression was markedly increased in high grade glioma (Grade IV and III), but there was no significant difference between low grade glioma (Grade II) and non-tumor brain tissues (Fig. 1a). Moreover, analysis of TCGA dataset showed significant increase of SKA1 expression in grade IV glioma compared with those in grade III glioma and grade II glioma (Fig. 1b). In brief, analysis of public dataset revealed that SKA1 expression was positively correlated with glioma grade in mRNA level. To further confirm these results, we examined the expression of SKA1 at protein level with tissue samples collected from Nanfang hospital, including glioma tissues (grade II, n = 5; grade III, n = 8; grade IV, n = 34) and non-tumor brain tissues (n = 5) with Western blot (Fig. 1c, d). Consistent with the results described above, significantly higher expression level of SKA1 was detected in Grade IV glioma.

**Fig. 1:** Increased SKA1 expression level was detected in glioma tissues and associated with poor prognosis in glioma. **a** In GEO dataset, the expression of SKA1 was markedly increased in high grade glioma (grade IV, n = 74; grade III, n = 30), but insignificantly different in low grade glioma (grade II, n = 44) compared with non-tumor brain tissues (n = 22). **b** In TCGA database, SKA1 expression was increased in grade IV glioma (n = 166), followed by grade III glioma (n = 259) and grade II glioma (n = 241). **c**, **d** Western blot analysis of glioma and non-tumor brain tissues collected from Nanfang hospital, the expression of SKA1 were positively correlated with WHO grades, β-actin was used as a loading control. **e** ROC curve showed the sensitivity and specificity of SKA1 as a biomarker to distinguish between glioblastoma and non-glioblastoma patients. **f**–**h** Kaplan–Meier analysis for overall survival (TCGA, n = 673; CGGA, n = 325) and progression-free survival (TCGA, n = 275) in glioma patients according to SKA1 expression level (*P *< 0.0001, by the log-rank test). Error bars represent the mean with extremum. *NB* non-tumor brain tissues

### SKA1 could serve as a potential diagnosis biomarker for GBM

Considering that SKA1 was overexpressed in grade IV glioma, we used Chinese Glioma Genome Atlas (CGGA) dataset to determine whether SKA1 could be used as a biomarker to distinguish between GBM and non-GBM patients (Grade II and III). The area under the receiver operating characteristic (ROC) curve of SKA1 for differential diagnosis was 0.774 (95% CI 0.716–0.832), indicating that SKA1 could serve as an effective diagnosis marker to distinguish glioblastoma patients from non-GBM patients (Grade II and III) (Fig. 1e).

### SKA1 overexpression was correlated with poor prognosis in glioma

In TCGA database, we observed that higher SKA1 expression was associated with worse overall survival (OS) and progression free survival (PFS) (Fig. 1f, g). The median OS in patients with higher SKA1 expression was 32.90 months compared with 95.83 months in those with lower expression (P < 0.0001). The median PFS of glioma patients with higher and lower expression of SKA1 was 10.27 months and 38.47 months, respectively (P < 0.0001). Consistently, SKA1 overexpression was also confirmed to be associated with worse OS in CGGA database (Fig. 1h).

### Suppression of SKA1 attenuated the cell viability in glioma cells in vitro and in vivo

To assess the function of SKA1 in glioma, three different lentiviral shRNA targeting SKA1 were used to specifically and stably knock down the SKA1 expression in four glioma cell lines including U87, U251, LN229 and T98. Among these three lentiviral particles, the most efficient shRNA vector, sh-SKA1-3, was confirmed with Western blot analysis and selected for further experiments (Fig. 2a).

**Fig. 2:** Suppression of SAK1 attenuates the proliferation ability of glioma cells in vitro. **a** U87, U251, LN229 and T98 cells were transfected with three shRNA vectors against SKA1, and knockdown efficiency were assessed with Western bolt. β-actin served as a loading control. Error bars represent the mean ± SD for three independent experiments (*P < 0.05). **b** Cell viability of U87 and U251 cells transfected with PLV-Ctr and shSKA1 was evaluated with CCK8 assay, respectively (*P < 0.05). **c** After SKA1 knockdown, fewer U87 and U251 cells were in S phase as shown in the EdU (red) assay. Nuclei were stained with DAPI (blue). **d** Proliferation ability of U U87 and U251 cells transfected with PLV-Ctr and shSKA1 was assessed with colony forming assay. Error bars represent the mean ± SD for three independent experiments (*P < 0.05)

CCK8 assays were subsequently performed to evaluate the effect of SKA1 on cell viability. After knockdown of SKA1, both U87 and U251 showed a slower rate of proliferation compared with the control group (Fig. 2b). The EdU incorporation assay revealed that the percentage of cells in S phase decreased after SKA1 knockdown in U87 and U251 cells (Fig. 2c). The results of colony forming assay performed in U87, U251, LN229 and T98 glioma cells further confirmed that suppression of SKA1 expression attenuated cell viability and proliferation of glioma cells in vitro (Fig. 2d).

To validate this result in vivo, subcutaneous xenograft tumor model was established in nude mice, which were divided into NC group and shSKA1 group with 10 mice per group. Mice were sacrificed at 30 days after tumor inoculation, and the average tumor weight was 0.925 g and 0.360 g, respectively (Fig. 3a, P < 0.0001). Furthermore, immunochemistry staining for the proliferation marker, PCNA, indicated that suppression of SKA1 significantly inhibited glioma proliferation in vivo (Fig. 3b, c).

**Fig. 3:** Suppression of SKA1 expression inhibited tumorigenicity of glioma cells in vivo. **a** When compared with PLV-Ctr group, tumorigenicity of shSKA1-U87 cells was markedly reduced in vivo (*P < 0.05). **b**, **c** Representative IHC images of N-Cadherin, E-Cadherin, MMP9 and PCNA staining in subcutaneous xenografts derived from indicated cells. Graphic representation scoring of indicated biomarkers expression (*P < 0.05). Original magnification ×400

### Suppression of SKA1 inhibited migration and invasion of glioma cells in vitro and in vivo

To examine the effect of SKA1 on glioma cell migration and invasion, Transwell assay, wound healing assay and Boyden assay were then performed. In Transwell assay, knockdown of SKA1 significantly decreased the percentage of migrated cells in the shSKA1 group (Fig. 4a), consistent with that found in wound healing assay (Fig. 4b). Additionally, Boyden assay revealed that SKA1 knockdown significantly suppressed the invasion of glioma cells (Fig. 4c). These results demonstrated that inhibition of SKA1 could significantly suppressed both migration and invasion of glioma cells in vitro. In xenograft models, we confirmed that knockdown of SKA1 could led to decreased N-cadherin and MMP9 and increased E-cadherin in xenograft tumor tissue (Fig. 3b, c).

**Fig. 4:** Suppression of SKA1 inhibits glioma cell migration and invasion ability in vitro. **a**, **b** Transwell and wound healing assay showed that SKA1 knockdown inhibited migration ability of glioma cell lines in vitro. **c** Boyden assay indicated that SKA1 knockdown significantly inhibited invasion ability of glioma cells in vitro. All values shown are mean ± SD of triplicate measurements (*P < 0.05)

### SKA1 regulated the expressions of cell cycle and EMT related proteins in glioma

To provide further insights into the mechanisms of SKA1 regulation, we used GSEA to investigate the possible biological functional of SKA1 in glioma with public dataset, including TCGA database and GEO dataset. GSEA results showed that SKA1 might be involved in cell cycle phase transition in glioma (Fig. 5a). Consistently, significantly decreased expressions of several cell cycle regulators and markers, such as FOXM1, CCNI, CCND1 and CDK1, were observed after SKA1 knockdown (Fig. 5b).

**Fig. 5:** SKA1 regulated cell cycle, EMT and Wnt/β-catenin signaling pathways in glioma cells. **a** Gene set enrichment analysis (GSEA) showed that there was a clear correlation between SKA1 expression and the cell cycle phase transition signature. **b** Expression of several cell cycle regulators and markers including FOXM1, CCNI, CCND1 and CDK1 was assessed with Western blot in U87 and U251 glioma cells with indicated treatments. **c** Expression of EMT-related and invasion-associated proteins including N-Cadherin, E-Cadherin, PLOD2, MMP2, Snail and Claudin were assessed with Western blot in U87 and U251 glioma cells with indicated treatments. **d** GSEA revealed SKA1 expression was associated with the Wnt-β-catenin signaling signature. **e** Expression of β-catenin and canonical Wnt/β-catenin signaling targets including CD44, c-Jun and c-Myc was examined with Western blot in U87 and U251 glioma cells with indicated treatments. All values were represented as mean ± SD of triplicate experiments (*P < 0.05)

Considering that IHC staining of xenograft tumors showed decreased N-cadherin and MMP9 under SKA1 inhibition, we then examined the effect of SKA1 knockdown on the expression of epithelial–mesenchymal transition (EMT) markers in vitro. Results showed that expression level of E-cadherin and Claudin was increased, and that of N-cadherin, PLOD2, MMP2 and Snail was significantly decreased after SKA1 knockdown in glioma cells (Fig. 5c).

### SKA1 also regulated Wnt/β-catenin signaling pathway

Additionally, GSEA results also indicated that SKA1 might be involved in Wnt/β-catenin signaling pathway. GSEA analysis of both RNA-seq and microarray dataset indicated that genes involved in Wnt/β-catenin signaling were enriched in glioma tissues with high expression of SKA1 (Fig. 5d). Consistently, with Western blot, significantly decreased expression level of β-catenin, and canonical Wnt/β-catenin signaling targets including CD44, c-Jun and c-Myc were observed under SKA1 inhibition (Fig. 5d).

## Discussion

In the present study, we identified SKA1 as a potential biomarker of malignant phenotype for glioma and confirmed that SKA1 expression increased along with advances of glioma grades. Based on these findings, we further investigated the biological functions of SKA1 in glioma and figured out that it could significantly promote glioma cells proliferation, migration and invasion abilities. With Western blot, we suggested that SKA1 may facilitate cell growth by regulation of cell cycle phase transition, contrary to that reported previously [17]. Finally, we demonstrated that SKA1 may also be involved in the regulation of EMT and Wnt/β-catenin signaling pathways.

Though SKA1 is firstly identified as a regulator of timely anaphase onset [9], recent oncology researches revealed that SKA1 may be a crucial regulator for tumorigenesis and multidrug-resistance in several tumors. Inhibition of SKA1 led to cell cycle arrest and apoptosis in a number of tumors including hepatocellular carcinoma, non-small cell lung carcinoma and gastric cancer [10, 15, 16]. SKA1 is also reported to be involved in chemo-resistance and contributes to cisplatin resistance in non-small cell lung carcinoma cells by protecting tumor cells from cisplatin-induced cell apoptosis [19]. Nevertheless, knockdown of SKA1 could sensitize tumor cells to tyrosine kinase inhibitor and epirubicin [13, 20].

Though precise regulatory network of SKA1 remains to be elucidated, several researches proposed that SKA1 could inhibit the activity of Akt and Erk pathway [21, 22]. Our manuscript reported the first evidence that SKA1 may also be involved in Wnt/β-catenin signaling pathway. Wnt/β-catenin signaling pathways is considered to be a fundamental growth control pathway, and its dysregulation is frequently observed in a variety of cancers, leading to a defined cellular response through the activation of β-catenin/TCF target genes [23]. It has been suggested that relative change rather than absolute change of β-catenin levels is crucial, indicating that even low levels of nuclear β-catenin are sufficed for target gene activation [24]. Since Wnt/β-catenin signaling pathway is involved in stemness and proliferative potential in several cancers [25–28], further work is needed to unravel potential involvement of SKA1 in glioma stemness.

## Conclusions

In conclusion, SKA1 expression increased along with advances of glioma grades, and SKA1 is a potential biomarker of poor prognosis for glioma. Particularly, SKA1 promotes proliferation, migration and invasion abilities in glioma cells. Furthermore, it is demonstrated that knockdown of SKA1 led to cell-cycle arrest and MET in glioma. Finally, we suggested that SKA1 could be a potential regulator of Wnt/β-catenin signaling pathway. Considering these results, SKA1 could a promising therapeutic target for the treatment of human glioma.

## Data Availability

The datasets analyzed in the current study were available from the corresponding author on reasonable request.

## Abbreviations

SKA1: spindle and kinetochore associated protein 1
EMT: epithelial–mesenchymal transition
MMP9: matrix metallopeptidase 9
PCNA: proliferating cell nuclear antigen
NB: non-tumor brain tissues
MET: mesenchymal–epithelial transition
